The article "ATF4 is a novel regulator of MCP-1 in microvascular endothelial cells" was published in 2015. Journal: J Inflamm (Lond).

# ATF4 is a novel regulator of MCP-1 in microvascular endothelial cells

**DOI:** 10.1186/s12950-015-0076-1

**Published:** 2015-04-17

**Authors:** Huibin Huang, Guangjun Jing, Joshua J Wang, Nader Sheibani, Sarah X Zhang

**Affiliations:** Departments of Ophthalmology and Biochemistry, School of Medicine and Biomedical Sciences, University at Buffalo, The State University of New York, Buffalo, NY 14214 USA; SUNY Eye Institute, The State University of New York, Buffalo, NY 14214 USA; Department of Medicine, Endocrinology and Diabetes, Harold Hamm Diabetes Center, University of Oklahoma Health Sciences Center, Oklahoma, 73104 OK USA; Department of Ophthalmology and Visual Sciences, University of Wisconsin, School of Medicine and Public Health, Madison, Wisconsin USA; McPherson Eye Research Institute, University of Wisconsin, School of Medicine and Public Health, Madison, WI 53705 USA; Department of Endocrinology, The 2nd Affiliated Hospital of Fujian Medical University, Quanzhou, Fujian China

**Keywords:** Monocyte chemoattractant protein 1, Microvascular endothelial cells, Activating transcription factor 4

## Abstract

**Background:**

Monocyte chemoattractant protein-1 (MCP-1) is a major chemokine that recruits monocyte/macrophage to the site of tissue injury and plays a critical role in microvascular complications of diabetes. However, the mechanisms underlying the regulation of MCP-1 are not fully understood. The present study aims to explore the role of activating transcription factor 4 (ATF4), an ER stress-inducible transcription factor, in regulation of MCP-1 expression and production in brain and retinal microvascular endothelial cells.

**Methods:**

For *in vitro* study, primary brain microvascular endothelial cells isolated from ATF4 knockout mice or mouse retinal endothelial cells were treated with lipopolysaccharide (LPS) to induce MCP-1 expression. ATF4 expression/function was manipulated by adenoviruses expressing wild type ATF4 (Ad-ATF4) or a dominant negative mutant of the protein (Ad-ATF4DN). For *in vivo* study, MCP-1 expression was induced by intravitreal injection of LPS or Ad-ATF4 in heterozygous ATF4 knockout or wild type mice.

**Results:**

LPS treatment induced a dose- and time-dependent increase in ATF4 expression, ER stress and MCP-1 production in brain and retinal microvascular endothelial cells. Overexpression of ATF4 in endothelial cells significantly increased the secretion of MCP-1 and promoted THP-1 monocyte-endothelial cell adhesion. Conditioned medium from ATF4-overexpressiing endothelial cells significantly enhanced THP-1 cell migration. Consistently, intravitreal injection of Ad-ATF4 remarkably enhanced retinal levels of MCP-1 and promoted inflammatory cell infiltration into the vitreous and retina. In contrast, LPS-induced MCP-1 upregulation was markedly attenuated in ATF4-deficient endothelial cells and in retinas of ATF4 knockout mice, suggesting that ATF4 is essential for LPS-induced MCP-1 production in endothelial cells and in the retina. Mechanistically, overexpression of ATF4 enhanced, while inhibition of ATF4, attenuated the basal and LPS-stimulated phosphorylation of NF-κB, P38, and JNK. Furthermore, pharmacological inhibition of NF-κB, P38, or JNK significantly reduced ATF4-stimulated MCP-1 secretion from endothelial cells.

The article "ATF4 is a novel regulator of MCP-1 in microvascular endothelial cells" was published in 2015. Journal: J Inflamm (Lond).

**Conclusions:**

Taken together, our results suggest a critical role of ATF4 in the regulation of MCP-1 production in retinal and brain microvascular endothelial cells, which may contribute to inflammation-related endothelial injury in diseases such as diabetic retinopathy.

## Background

The endoplasmic reticulum (ER) is the central hub for protein biosynthesis, protein folding and regulation of intracellular calcium concentration. A delicate balance between protein synthesis and folding is vital for cell survival and function. However, this homeostasis can be disturbed in some physiological or pathophysiological conditions, due to increased demand of protein production, reduced capacity of protein folding, altered redox status in the ER, or perturbed protein and calcium trafficking [1]. As a consequence, unfolded or misfolded proteins accumulate in the ER, resulting in activation of the unfolded protein response (UPR) by three ER membrane proteins: inositol requiring trans-membrane kinase/endonuclease 1 (IRE1), activating transcription factor 6 (ATF6) and protein kinase (PKR)-like endoplasmic reticulum kinase (PERK). PERK, through phosphorylation of eukaryotic translation initiation factor 2α (eIF2α), suppresses global protein translation but increases the production of activating transcription factor 4 (ATF4), inducing the expression of C/EBP homologous protein (CHOP) [2]. Chronic ER stress results in apoptosis and cell death, contributing to retinal degeneration [3]. In addition, our recent studies have shown that ER stress and the PERK/eIF2α/ATF4/CHOP pathway are involved in regulation of immune response and retinal vascular injury in diabetic retinopathy, a common complication of diabetes [4,5]. However, the mechanisms underlying ER stress-related inflammatory signaling are not fully understood.

The innate immune system is a critical component of host defense, which recognizes pathogen-associated molecules through pathogen-recognition receptors, such as Toll-like receptors (TLRs) [6]. TLR4 recognizes specific structural components of pathogens, such as lipopolysaccharide (LPS), resulting in the activation of MyD88-dependent and TRIF-dependent pathways. The MyD88-dependent pathway primarily activates signaling proteins including TGF-beta-activated kinase (TAK)-nuclear factor (NF)-κB and TAK-mitogen-activated protein kinase (MAPK)-AP-1[7]. The activation of these transcription factors induces the expression of multiple pro-inflammatory factors, such as monocyte chemoattractant protein-1 (MCP-1). Intriguingly, several studies have revealed a role of ER stress and the UPR in regulation of the TLR signaling [8,9]. In macrophages, induction of the UPR acts synergistically with LPS in production of cytokines such as interleukin 23 and interleukin 17 [10,11]. Moreover, activation of ATF4 has been shown to promote the secretion of interleukin 6, interleukin 8 and RANTES through an interaction with c-Jun of the TLR4-MyD88 pathway. Paradoxically, recent work by Woo and colleagues indicates that pretreatment with low dose of LPS selectively suppresses the PERK-ATF4-CHOP pathway [12] and protects mice from tunicamycin-induced renal dysfunction and hepatosteatosis [12]. These findings indicate some complex interactions between the UPR and TLR4 signaling, which may contribute to the tight control of inflammatory factor expression during tissue injury.

The article "ATF4 is a novel regulator of MCP-1 in microvascular endothelial cells" was published in 2015. Journal: J Inflamm (Lond).

In diabetic retinopathy, increased MCP-1 production is a major factor responsible for leukocyte migration and interaction with endothelium resulting in microvascular injury of the retina. Previously we have shown that ATF4 was upregulated in diabetic retina and was required for pro-inflammatory genes VEGF (vascular endothelial growth factor) and ICAM-1 (intercellular adhesion molecule 1) expression in Müller and vascular endothelial cells [4,5]. In the present study, we investigated the role of ATF4 in MCP-1 production from brain and retinal microvascular endothelial cells and explored the underlying mechanisms by which ATF4 regulates MCP-1 expression.

## Materials and methods

### Materials

Thapsigargin (TG) was obtained from Sigma-Aldrich (St. Louis, MO). JNK inhibitor II (SP600125), P38 inhibitor (SB203580), and p44/42 inhibitor (U0126) were purchased from Calbiochem (San Diego, CA). NF-κB inhibitor (Ro106-9920) was obtained from Tocris Bioscience. Endothelial cell growth supplement kit was obtained from Millipore (Billerica, MA). Protease inhibitor cocktail, anti-ATF4, anti-CHOP, antibodies were purchased from Santa Cruz Biotechnology (Santa Cruz, CA). Anti-phospho-eIF2α, anti–eIF2α, anti-phospho-JNK, anti- phospho-P38, anti-phospho-NF-κB, and anti- phospho-p44/42 antibodies were obtained from Cell Signaling (Danvers, MA), and anti-β-actin antibody was from Abcam (Cambridge, MA). Horseradish peroxidase–conjugated, fluorescein isothiocyanate avidin (FITC)-conjugated, or biotinylated secondary antibodies, and DAPI were purchased from Vector Laboratories (Burlingame, CA). Cy3-conjugated anti-rabbit IgG was obtained from Jackson ImmunoResearch Laboratories (West Grove, PA).

The article "ATF4 is a novel regulator of MCP-1 in microvascular endothelial cells" was published in 2015. Journal: J Inflamm (Lond).

### Cell culture

Immortalized mouse retinal endothelial cells [13] were grown at 33°C in DMEM with 10% FBS and 30 μg/ml endothelial cell growth supplement. THP-1 cells were obtained from ATCC (Manassas, VA) and were routinely maintained in RPMI 1640 medium with 10% fetal bovine serum and 0.05 mM 2-mercaptoethanol. Mouse brain microvascular endothelial cells were isolated as described previously [14] and were grown in DMEM with 20% FBS. To better recapitulate the *in vivo* situation and to reduce the confounding effects of the serum, subconfluent cells were starved with DMEM containing 1% FBS to acquire quiescence prior to the desired treatments.

### Experimental animals

C57BL/6 J mice were purchased from the Jackson Laboratory (BarHarbor,ME). ATF4 knockout mice were kindly provided by Tim Townes, Ph.D. (University of Alabama at Birmingham) [4,5]. Care, use, and treatment of all animals were in strict agreement with the guidelines of the Association for Research in Vision and Ophthalmology Statement for the Use of Animals in Ophthalmic and Visual Research and approved by the institutional animal care and use committees in the University of Oklahoma Health Sciences Center.

### Intravitreal injection of adenovirus

Intravitreal injection was performed in deeply anesthetized mice using an UltraMicroPump (World Precision Instruments, Sarasota, FL). Briefly, an incision was made 1 mm behind the limbus with a sharp-edge 31-gauge needle. The 34-gauge blunt needle mounted on a 10-μl microsyringe was inserted into the vitreous cavity. One microliter of vehicle containing 10^9^ viral particles was delivered into the vitreous with one foot-switch press.

### Transduction of microvascular endothelial cells with adenovirus

Adenoviruses expressing wild-type ATF4 (Ad-ATF4) or a dominant negative mutant of ATF4 (Ad-ATF4DN) were generated and propagated as described previously [4,5]. Empty adenoviruses that did not contain a transgene were used as control. Retinal or brain microvascular endothelial cells were transduced with adenoviruses at 30 MOI (multiplicity of infection) (for immortalized mouse retinal endothelial cells) or 100 MOI (for primary mouse brain endothelial cells) for 24 h. Cells were then exposed to DMEM containing 1% FBS overnight to acquire quiescence prior to the desired treatments.

### Histology and immunofluorescence

For retinal histological study, eyeballs were immersed in Per-fix (4% paraformaldehyde, 20% isopropanol, 2% trichloroacetic acid, 2% zinc chloride) overnight and embedded in paraffin. Sagittal sections of 5 μm thickness were stained with hematoxylin and eosin (HE) and examined under an Olympus microscopy (Tokyo, Japan). Immunofluorescence study on retinal cryosections was prepared as previously described [11]. Briefly, the sections were immunostained with anti-CD11b antibody (1:100 dilution) overnight at 4°C. Negative controls without primary antibody incubation were included. After multiple washes, the sections were incubated with Cy3-conjugated secondary antibody (Molecular Probes, Eugene, OR, USA). DAPI was used to label cell nuclei.

The article "ATF4 is a novel regulator of MCP-1 in microvascular endothelial cells" was published in 2015. Journal: J Inflamm (Lond).

### Real-time qPCR

Total RNA was extracted using the RNeasy Mini Kit (Qiagen). cDNA was synthesized using the iScript cDNA Synthesis Kit, and Real-time qPCR was performed using SYBR Green PCR Master Mix (Bio-Rad Laboratories, Hercules, CA, USA) on an iCycler iQTM (BioRad, Hercules, CA). Relative mRNA level was calculated by the ΔΔCt method and ribosomal protein L19 (Rlp19) was used as an endogenous control. The sequences of primers for mouse MCP-1 are as following: forward: ATGAGATCAGAACCTACAACT; reverse: TCCTACAGAAGTGCTTGAG.

### Transwell migration assay

The transwell migration assay was performed on semi-permeable membranes with pore size of 5 μm (Costar Transwell, Corning, NY). Briefly, THP-1 cells were suspended in RPMI1640 medium supplemented with 1% FBS and 0.5% BSA (Sigma-Aldrich). 1 × 10^5^ cells were seeded in the transwell inserts and allowed to migrate overnight toward the lower compartments with the conditioned medium from endothelial cell culture. The membranes of the inserts were fixed with 4% paraformaldehyde. Cells on the top surface of the membrane were mechanically removed, and those migrated to the bottom of the membrane were stained with DAPI (4’, 6- diamidino-2-phenylindole). Cell numbers were counted in 3 random visual fields, using an Olympus fluorescence microscope (Tokyo, Japan).

### Leukocyte adhesion assay

Endothelial cells were grown to 80% confluence in six-well plates and pretreated with LPS or Ad-ATF4 with controls for 24 h. THP-1 cells were added to endothelial culture and incubated for additional 3 h. Unbound THP-1 cells were removed by 3 washes with PBS, and bound THP-1 monocytes were counted from 3 random visual fields under an Olympus microscope (Tokyo, Japan).

### Western blot analysis

Cells or retina tissue were lysed in radioimmunoprecipitation assay lysis buffer (RIPA, Santa Cruz). Western blot analysis was performed as described previously [4,5]. The following primary antibodies were used at the indicated dilutions: anti-phospho-eIF2α (1:1,000), anti-eIF2α (1:1,000), anti-ATF4 (1:500), anti-CHOP (1:500), anti-phospho-JNK (1:500), anti-phospho-p38 (1:1000), antiphospho-p44/42(1:1000), anti-phospho-NF-κB (1:1000), and anti-β-actin (1:5,000) antibodies. Horseradish peroxidase-conjugated goat-anti-rabbit IgG (Vector Laboratories, Bulingame, CA) and goat anti-mouse IgG (Vector Laboratories) were used as secondary antibodies.

The article "ATF4 is a novel regulator of MCP-1 in microvascular endothelial cells" was published in 2015. Journal: J Inflamm (Lond).

### ELISA

MCP-1 was quantified using mouse MCP-1 ELISA assay kit (R&D systems, Minneapolis, MN) according to manufacturer’s instructions.

### Statistical analysis

Statistical analysis was performed using Student’s t test when comparing two groups, or ANOVA with Bonferroni’s post hoc test when comparing three or more groups. Statistical significance was accepted as p < 0.05.

## Results

### LPS increases ER stress and ATF4 expression in microvascular endothelial cells

We first examined whether activation of the TLR4 signaling by LPS induces ER stress and ATF4 expression in mouse brain and retina microvascular endothelial cells. Our results show that 31.25 ng/mL to 500 ng/mL of LPS significantly increased ATF4 levels in a dose-dependent manner (Figure 1A). The maximal induction of ATF was observed in cells treated with 250 ng/ml of LPS. To determine the time course of ATF4 induction, cells were exposed to LPS (250 ng/ml) for 0–48 h. Western blot analysis shows that the levels of ATF4 increased at 12 h, continued to increase at 24 h, and slightly declined at 48 h (Figure 1A). In line with these changes, 24 h of LPS treatment significantly increased the levels of ATF4-related ER stress markers, including eIF2α phosphorylation and CHOP in both retinal (Figure 1B) and brain (Figure 1C) endothelial cells, and the inductions appeared to be more profound in brain endothelial cells than retinal endothelial cells. Moreover, LPS treatment markedly increased MCP-1 mRNA expression (Figure 1D) and protein secretion (Figure 1E). The temporal correlations suggest a potential role of ER stress and ATF4 in MCP-1 production in microvascular endothelial cells.

**Figure 1:** LPS increases ER stress and ATF4 expression in mouse microvascular endothelial cells. **A)**. Mouse retinal endothelial cells were treated with 31.25 ng/ml - 250 ng/ml of LPS for 24 h or treated with 250 ng/ml of LPS for 0–48 h. The levels of ATF4 were determined by western blot analysis and quantified by densitometry. **B)**. Mouse retinal endothelial cells were treated with 250 ng/ml of LPS for 24 h, the levels of phosphorylated and total eIF2α, ATF4, and CHOP were analyzed. **C)**. Mouse brain endothelial cells were treated with 250 ng/ml of LPS at for 8 h. The levels of phosphorylated and total eIF2α, ATF4, and CHOP were examined. **D-E)**. Mouse retinal endothelial cells were treated with 250 ng/ml of LPS for 24 h. The mRNA levels of MCP-1 were determined by qPCR **(D)**. The levels of MCP-1 in the medium were measured by ELISA **(E)**. Results were expressed as mean ± SD (n = 3). *P < 0.05, **P < 0.01, ***P <0.001 vs. control.

The article "ATF4 is a novel regulator of MCP-1 in microvascular endothelial cells" was published in 2015. Journal: J Inflamm (Lond).

### ATF4 mediates LPS-induced MCP-1 production in microvascular endothelial cells

Previously we have shown that ATF4 is required for the expression of two major pro-inflammatory genes, VEGF and ICAM-1, in retinal Müller and endothelial cells [4,5,15]. In order to elucidate if ATF4 mediates LPS-induced MCP-1 production from endothelial cells, gain-of-function and loss-of-function experiments were performed using adenoviruses expressing wild type ATF4 (Ad-ATF4) or its dominant negative form (Ad-ATF4DN). The efficiency of adenoviral transduction and protein expression in mouse retinal endothelial cells were confirmed in Figure 2A. Following viral transduction, cells were incubated with 250 ng/ml of LPS for 24 h. The levels of MCP-1 mRNA expression and protein secretion were measured by real-time PCR and ELISA, respectively. Our results show that overexpression of ATF4 resulted in a 2.8-fold increase in MCP-1 mRNA and significantly enhanced LPS-induced MCP-1 expression (Figure 2B). Inhibition of ATF4 did not alter the basal level of MCP-1 but reduced LPS-stimulated MCP-1 expression by 40% (Figure 2C). At protein level, treatment with Ad-ATF4 or LPS alone induced a 2-fold increase in MCP-1 secretion (Figure 2D). Combination of Ad-ATF4 and LPS increased MCP-1 secretion nearly 6 fold, indicating a synergistic effect of ATF4 and LPS in MCP-1 secretion. Inhibition of ATF4 activity reduced LPS-stimulated MCP-1 secretion by 37% (Figure 2D). In line with these results, brain endothelial cells isolated from ATF4 −/− mice showed a 40% reduction in MCP-1 secretion when challenged with LPS, compared to ATF4 +/+ endothelial cells (Figure 2E). Interestingly, overexpression of ATF4 induced a 4-fold increase in MCP-1 secretion in brain endothelial cells (Figure 2F). These results indicate that ATF4 is both sufficient and essential for LPS-induced MCP-1 production in microvascular endothelial cells.

**Figure 2:** ATF4 mediates LPS-induced MCP-1 production in mouse microvascular endothelial cells. **A-D)**. Mouse retina endothelial cells were transduced with Ad-ATF4, Ad-ATF4DN, or Ad-Ctrl for 24 h and then treated with 250 ng/ml of LPS for extra 24 h. The levels of MCP-1 mRNA expression and protein secretion were measured by qPCR or ELISA, respectively. **E)**. ATF4 +/+ or ATF4 −/− mouse brain endothelial cells were stimulated with 250 ng/ml of LPS for 8 h. MCP-1 secretion in the medium was evaluated by ELISA. **F)**. ATF4+/+ mouse brain endothelial cells were transduced with Ad-Ctrl or Ad-ATF4 and then treated with 250 ng/ml of LPS for 8 h. MCP-1 secretion was measured by ELISA. Results were expressed as mean ± SD. * P < 0.05, ** P < 0.01, *** p < 0.001 vs. Ad-Ctrl; ++ P < 0.01, +++ P < 0.001 vs. WT + LPS or Ad-Ctrl + LPS.

The article "ATF4 is a novel regulator of MCP-1 in microvascular endothelial cells" was published in 2015. Journal: J Inflamm (Lond).

### ATF4 regulates retinal MCP-1 expression and leukocyte infiltration *in vivo*

To confirm the *in vitro* results, we conducted two independent sets of experiments with wild type (WT) and heterozygous ATF4 knockout (KO) mice. As described previously, homozygous ATF4 KO mice are not suitable for eye experiment due to the defect in the development of the lens [4,5]. In the first experiment, 250 ng of LPS was injected into the vitreous cavity of one eye of a mouse and equal volume of PBS was injected into the contralateral eye as control. Retinal MCP-1 expression was determined by real-time qPCR at 24 h post-injection. Our results show that LPS induced over 20 fold increase in MCP-1 expression in WT mice and, to a significantly less extent (5 fold increase) in ATF4 KO mice (Figure 3A). In addition, the basal MCP-1 expression was reduced in the retina of ATF4 KO mice, suggesting ATF4 is essential for retinal MCP-1 expression in both static and stimulated conditions. In the second experiment, we overexpressed ATF4 in the retina by intravitreal injection of Ad-ATF4 in C57/BL6J mice. We found that overexpression of ATF4 resulted in a 3-fold increase in retinal MCP-1 production when compared to control (Figure 3B). Furthermore, we observed a large number of leukocytes accumulating in the vitreous and the retina, predominantly in the area around the optic nerve head, in the eyes injected with Ad-ATF4 (Figure 3C). These changes were further confirmed by increased expression of CD11b, a surface marker of leukocytes [16], in the retina after Ad-ATF4 treatment (Figure 3D). Taken together, these results suggest a critical role of ATF4 in LPS-induced retinal MCP-1 production and leukocyte infiltration.

**Figure 3:** ATF4 regulates retinal MCP-1 expression and leukocyte infiltration *in vivo*. **A)**. Wild type (WT) or heterozygous ATF4 knockout (KO) mice received intravitreal injection of 250 ng of LPS in one eye and PBS as control in the contralateral eye. Twenty-four hours after injection, retinal MCP-1 expression was determined by qPCR (n = 5). Results were expressed as mean ± SD. *P < 0.05 vs. WT + PBS; ++ P < 0.01 vs. WT + LPS. **B-D)**. C57/B6J mice received intravitreal injection of 1 μl of Ad-ATF4 or Ad-Ctrl (10^9^ viral particles). After 5 days, retinas were harvested and MCP-1 level was measured by ELISA **(B)**. Results are expressed as mean ± SD, n = 5. *P < 0.05 vs. Ad-Ctrl. Leukocyte infiltration into the vitreous and retina was analyzed by H&E staining of paraffin sections **(C)**. and immunofluorescence analysis for monocyte/macrophage marker CD11b **(D)**. GCL: ganglion cell layer, INL: inner nuclear layer, ONL: outer nuclear layer. Black arrows indicate inflammatory cell infiltration into the vitreous **(C)** and white arrows indicate CD11b positive cells in the retina **(D)**. Images were representative of 3 mice in each group.

The article "ATF4 is a novel regulator of MCP-1 in microvascular endothelial cells" was published in 2015. Journal: J Inflamm (Lond).

### Manipulating ATF4 expression in endothelial cells influences leukocyte migration and leukocyte-endothelial adhesion

MCP-1 is considered a key regulator of monocyte adhesion, migration and recruitment. We hypothesize that ATF4 regulates MCP-1 secretion from retinal endothelial cells, which in turn promotes monocyte/macrophage adhesion and migration into retinal tissue resulting in inflammation. To test this hypothesis, retinal and brain endothelial cells were transduced with Ad-ATF4 or treated with 250 ng/ml of LPS for 24 h. Conditioned medium was collected from endothelial culture and added to cultured THP-1 cells. After 24 h of incubation, THP-1 cells were subjected to migration assay. Results show that incubation with the conditioned medium from ATF4-overexpressing endothelial cells significantly enhanced THP-1 cell migration (Figure 4A). Likewise, incubation with the medium from LPS-challenged wild type (ATF4 +/+) endothelial cells also induced a robust increase in THP-1 cell migration. This effect was markedly reduced in the cells incubated with the medium from LPS-treated ATF4−/− endothelial cells (Figure 4B), suggesting that ATF4 is required for LPS-stimulated inflammatory factor secretion from endothelial cells. In contrast, conditioned medium from unstimulated ATF4 +/+ or ATF4 −/− endothelial cells had negligible effect on THP-1 migration.

**Figure 4:** Effects of conditioned medium derived from endothelial cells overexpressing or lacking ATF4 on THP-1 cell migration. **A)**. Mouse retinal endothelial cells were transduced with Ad-Ctrl or Ad-ATF4 for 24 h. **B)**. Brain endothelial cells isolated from ATF4 +/+ or ATF4 −/− mice were challenged with 250 ng/ml LPS for 24 h. The medium was collected from endothelial cell culture and used for THP-1 cell migration assay as described in the Method section. Left panels: representative images of migrated THP-1 cells (200×). Right panels: The numbers of migrated cells were quantified from 3 independent experiments. Results are expressed as mean ± SD (n = 3). ** P < 0.01 vs. Ad-Ctrl or WT; ++ p < 0.01 vs. WT + LPS.

The article "ATF4 is a novel regulator of MCP-1 in microvascular endothelial cells" was published in 2015. Journal: J Inflamm (Lond).

Next, we investigated whether manipulation of ATF4 expression in endothelial cells affects monocyte-endothelial adhesion. Prior to the adhesion assay, retinal endothelial cells were transduced with Ad-ATF4 or control adenovirus for 24 h. ATF4 +/+ or ATF4 −/− brain endothelial cells were pre-treated with LPS for 24 h. Endothelial-monocyte adhesion assay was performed as described in the Method section. Results show that overexpressing ATF4 in endothelial cells significantly increased monocyte-endothelial adhesion (Figure 5A). LPS treatment of ATF4 +/+ endothelial cells also resulted in an over 10-fold increase in THP-1 adhesion, which was markedly reduced in ATF4 −/− cells (Figure 5B). Unstimulated ATF4 +/+ and ATF4 −/− endothelial cells demonstrated similar capability in inducing THP-1 adhesion. These results strongly suggest a critical role of endothelial ATF4 in promoting monocyte migration and adhesion to endothelial cells.

**Figure 5:** Overexpressing/suppressing ATF4 in endothelial cells promotes/inhibits THP-1 cell adhesion. **A)**. Mouse retinal endothelial cells were transduced with Ad-Ctrl or Ad-ATF4 for 24 h. THP-1 cells were added and co-cultured for 3 hours. Adherent monocytes to endothelial cells were counted from 5 random visual fields. **B)**. Brain endothelial cells isolated from ATF4 +/+ or ATF4−/− mice were challenged with 250 ng/ml LPS for 24 h. THP-1 monocyte adhesion was assessed as described in **(A)**. Images are representatives of 3 independent experiments. Results are expressed as mean ± SD (n = 3). ** P < 0.01 vs. Ad-Ctrl or WT; ++ p < 0.01 vs. WT + LPS.

### ATF4 up-regulates MCP-1 through NF-κB and MAPK pathways

NF-κB and AP-1 are key transcription factors in LPS-activated TLR4/MyD88 pathway that upregulate inflammatory genes, such as MCP-1. To elucidate the mechanisms by which ATF4 promotes MCP-1 expression, we evaluated the effects of ATF4 on NF-κB and MAPK activation. In retinal endothelial cells, inhibition of ATF4 by Ad-ATF4DN significantly reduced both the basal and LPS-stimulated phosphorylation of NF-κB, P38, and JNK, but did not alter the phosphorylation of P44/42 (Figure 6A). In contrast, overexpression of ATF4 increased phosphorylation of NF-κB, P38 and JNK, but not P44/42 (Figure 6B). LPS treatment further enhanced phosphorylation of NF-κB and MAPKs, indicating a synergistic effect of LPS treatment and overexpression of ATF4 on activation of these pathways.

**Figure 6:** ATF4 is required for LPS-induced NF-κB and MAPK activation in retinal endothelial cells. Mouse retina endothelial cells were transduced with Ad-Ctrl, Ad-ATF4DN **(A)**, or Ad-ATF4 **(B)** for 24 h and then treated with 250 ng/ml LPS for additional 8 h. The levels of p-NF-κB, p-P38, p-JNK, p-P42/44 were determined by western blot analysis and quantified by densitometry. Results are expressed as mean ± SD (n = 3). * P < 0.05, ** P < 0.01 vs. Ad-Ctrl; + P < 0.05, ++ P < 0.01 vs. Ad-Ctrl + LPS.

The article "ATF4 is a novel regulator of MCP-1 in microvascular endothelial cells" was published in 2015. Journal: J Inflamm (Lond).

In brain microvascular endothelial cells, LPS induced a much less increase in NF-κB, P38 and JNK activation in ATF4–deficient cells (Figure 7A). These results have further confirmed the findings from retinal endothelial cells that inhibition of ATF4 reduces the activation of NF-κB, P38 and JNK pathways. To clarify the roles of NF-κB and MAPK pathways in ATF4-mediated MCP-1 upregulation, brain endothelial cells were pretreated with pharmacological inhibitors of NF-κB, P38, JNK, and P44/42 and then transduced with Ad-ATF4 or Ad-Ctrl. Pretreatment with inhibitors of NF-κB, P38, JNK, but not P44/42, significantly reduced MCP-1 secretion induced by Ad-ATF4 (Figure 7B). These results suggest that the activation of NF-κB, P38, and JNK is involved in ATF4-induced MCP-1 production.

**Figure 7:** ATF4 regulates MCP-1 expression through enhancing NF-κB and MAPK activation. **A)**. Brain endothelial cells from ATF4 +/+ and ATF4 −/− mice were treated with 250 ng/ml LPS for 8 h. The levels of p-NF-κB, p-P38, p-JNK, p-P42/44 were determined by western blot analysis and quantified by densitometry (mean ± SD, n = 3). *P < 0.05 vs. WT; +P < 0.05, ++P < 0.01 vs. WT + LPS. **B)**. Brain endothelial cells from ATF4 +/+ mice were pretreated with 1 μM Ro106, 10 μM SB203580, 10 μM SP600125 or 10 μM U0126 for 1 h, followed by transduction with Ad-ATF4 or Ad-Ctrl for 24 h. MCP-1 protein levels in the media were measured by ELISA. Results are expressed as mean ± SD (n = 3). ** P < 0.01 vs. Ad-Ctrl; + P < 0.05, ++ P < 0.01 vs. Ad-ATF4.

## Discussion

We have previously shown that ATF4 is involved in the regulation of inflammatory genes in retinal endothelial and Müller cells [4,5]. However, the mechanisms are not fully defined. Herein, we demonstrate that ATF4 is essential for MCP-1 expression in endothelial cells, likely through promoting the activation of NF-κB and MAPK pathways. ATF4 is a major stress response gene activated in cells under conditions of ER stress and oxidative stress [4,5,17-20]. As a transcription factor, ATF4 regulates a variety of genes involved in multiple biological processes, including hematopoiesis, lens and skeletal development, inflammation, angiogenesis, oxidative stress, and apoptosis. Recently studies suggest that ATF4 is up-regulated in various pathogen-induced-immune responses and participates in the TLR signaling pathways [12,21-23]. Coincidently, other UPR branches are also activated, reflecting the concurrence of ER stress with ATF4 activation [24-29]. Moreover, activation of ATF4 enhances TLR4-induced secretion of pro-inflammatory cytokines (IL-6 and IL-8) in macrophages [30]. In line with these findings, we show that activation of TLR4 by LPS induces ER stress and upregulates ATF4 in brain and retinal microvascular endothelial cells. Over-expression of ATF4 was sufficient to induce MCP-1 expression. In contrast, inhibition of ATF4 significantly attenuated LPS-induced MCP-1 secretion. These observations support our previous findings that ATF4 is an important regulator of retinal inflammatory response and vascular leakage in diabetic retinopathy [5] and further reveals a role of MCP-1 in ATF4-mediated retinal inflammation.

The article "ATF4 is a novel regulator of MCP-1 in microvascular endothelial cells" was published in 2015. Journal: J Inflamm (Lond).

MCP-1 is a key chemokine that regulates monocyte/macrophage migration and recruitment in inflammatory tissues [31-34]. Herein, we provided several lines of evidence that support a critical role of ATF4 in regulation of MCP-1 production and inflammatory cell infiltration. First, we found the MCP-1 level was increased in the medium from ATF4-overexpressing endothelial cells, and both adhesion and migration of THP-1 cells were enhanced when incubated with this conditioned medium. Second, using the medium from ATF4-deficient endothelial cells impaired monocyte adhesion and migration, even in the presence of LPS. A limitation of these experiments is using THP-1 cells, a human monocyte cell line, to investigate adhesion to murine endothelial cells. Although THP-1 cells have been extensively used for adhesion and migration assays, future studies using murine J774 cells to confirm the results from the current study is necessary. Third, over-expression of ATF4 *in vivo* promoted macrophage infiltration into the vitreous and retina. These findings indicate that ATF4 is involved in MCP-1 regulation in endothelial cells, which in turn modulates monocyte/macrophage activity and retinal inflammatory response. It is notable that although MCP-1 is abundant in the endothelial culture supernatant, there are likely other secreted factors that are regulated by ATF4 and contribute to macrophage migration. Future studies to eliminate or deactivate MCP-1 protein by applying a neutralising antibody against MCP-1 to the conditioned medium or using supernatant from MCP1-null endothelial cells engineered to overexpress ATF4 are warranted to clarify the role of MCP-1 in mediating the effect of ATF4 upregulation in endothelial cells on macrophage adhesion and infiltration.

LPS activation of the TLR4 signaling, through MyD88-downstream NF-κB and AP-1 pathways, leads to the induction of pro-inflammatory cytokines including MCP-1 [35,36]. Recent studies found that upon LPS stimulation, ATF4 forms dimer with JNK via the AP-1 and CREB binding sites, promoting the secretion of various pro-inflammatory cytokines in human monocytes/macrophages [30]. Our previous work also indicates a crosstalk between ATF4 and classic inflammatory signals including STAT3 and JNK in retinal endothelial and Müller cells, respectively [4,5]. Now, we demonstrate that deletion of ATF4 or inhibition of ATF4 function significantly attenuates the basal and LPS-stimulated phosphorylation of NF-κB, P38, and JNK. In contrast, overexpressing ATF4 is sufficient to activate these signaling molecules, which are required for ATF4-mediated MCP-1 expression. These results have revealed a new mechanism by which ATF4 interacts with TLR4 pathways through activation of MyD88 downstream effectors and, thus, might be a central coordinator for inflammatory response in microvascular endothelial cells in the brain and the retina.

The article "ATF4 is a novel regulator of MCP-1 in microvascular endothelial cells" was published in 2015. Journal: J Inflamm (Lond).

## Conclusions

Our data suggest that ATF4 functions as a positive regulator in LPS-triggered MCP-1 production in endothelial cells through multiple pathways. This mechanism could reveal a new target in endothelial cells to prevent vascular pathology associated with monocyte/macrophage-mediated inflammation in diseases such as diabetic microvascular complications.
